The article "Associations of TGFBR1 and TGFBR2 gene polymorphisms with the risk of hypospadias: a case–control study in a Chinese population" was retracted in 2022. Reasons: false authorship; concerns about the authorship.

# Associations of TGFBR1 and TGFBR2 gene polymorphisms with the risk of hypospadias: a case–control study in a Chinese population

**DOI:** 10.1042/BSR20170713

**Published:** 2017-10-06

**Authors:** Xin-Rui Han, Xin Wen, Shan Wang, Xiao-Wu Hong, Shao-Hua Fan, Juan Zhuang, Yong-Jian Wang, Zi-Feng Zhang, Meng-Qiu Li, Bin Hu, Qun Shan, Chun-Hui Sun, Ya-Xing Bao, Meng Lin, Tan He, Dong-Mei Wu, Jun Lu, Yuan-Lin Zheng

**Affiliations:** 1 Key Laboratory for Biotechnology on Medicinal Plants of Jiangsu Province, School of Life Science, Jiangsu Normal University, Xuzhou 221116, P.R. China; 2 Department of Immunology, School of Basic Medical Sciences, Fudan University, Shanghai 200032, P.R. China; 3 Jiangsu Key Laboratory for Eco-Agricultural Biotechnology around Hongze Lake, School of Life Sciences, Huaiyin Normal University, Huaian 223300, P.R. China; 4 Department of Orthopedics, The Affiliated Municipal Hospital of Xuzhou Medical University, Xuzhou 221009, P.R. China; 5 Department of Urology Surgery, Peking Union Medical College Hospital, Beijing 100730, P.R. China

**Keywords:** Gene polymorphism, Hypospadias, Case-control, Risk, TGFBR1, TGFBR2

## Abstract

This case–control study investigated the association of transforming growth factor-β (TGF-β) receptor type I and II (*TGFBR1* and *TGFBR2*) gene polymorphisms with the risk of hypospadias in a Chinese population. One hundred and sixty two patients suffering from hypospadias were enrolled as case group and 165 children who underwent circumcision were recruited as control group. Single nucleotide polymorphisms (SNPs) in *TGFBR1* and *TGFBR2* genes were selected on the basis of genetic data obtained from HapMap. PCR-restriction fragment length polymorphism (PCR-RFLP) was performed to identify TGFBR1 and TGFBR2 gene polymorphisms and analyze genotype distribution and allele frequency. Logistic regression analysis was conducted to estimate the risk factors for hypospadias. No significant difference was found concerning the genotype and allele frequencies of TGFBR1 rs4743325 polymorphism between the case and control groups. However, genotype and allele frequencies of TGFBR2 rs6785358 in the case group were significantly different in contrast with those in the control group. Patients carrying the G allele of TGFBR2 rs6785358 polymorphism exhibited a higher risk of hypospadias compared with the patients carrying the A allele (*P*<0.05). The TGFBR2 rs6785358 genotype was found to be significantly related to abnormal pregnancy and preterm birth (both *P*<0.05). The frequency of TGFBR2 rs6785358 GG genotype exhibited significant differences amongst patients suffering from four different pathological types of hypospadias. Logistic regression analysis revealed that preterm birth, abnormal pregnancy, and TGFBR2 rs6785358 were the independent risk factors for hypospadias. Our study provides evidence that TGFBR2 rs6785358 polymorphism might be associated with the risk of hypospadias.

## Introduction

Hypospadias is a highly common congenital abnormality in the male external genitalia occurring in every 4–6 male newborns per 1000, and especially rising in the last 30 years [1]. In newborn males, hypospadias is the second most common congenital anomaly after undescended testis [2]. Hypospadias can be classified into distal, medial, and proximal subtypes according to the position of the urethral opening; besides, for patients suffering from proximal hypospadias, they may be scrotal, perineal, and penoscrotal hypospadias [3]. Hypospadias surgery has been widely used in the region of urogenital reconstructive surgery using various techniques; for example the two-stage repair is a favorable method for proximal hypospadias [4]. The multifarious etiology of hypospadias remains unknown but seems to be an integration of genetic susceptibility, environmental pollutants, a maternal diet lacking protein, placental insufficiency, the use of hormone-containing contraceptives post-conception, high maternal BMI, parental subfertility, and endocrine disruption [5–10]. Hence, it is urged to acquire a full-scale knowledge of genetic mutations in the development of hypospadias.

Single nucleotide polymorphisms (SNPs) in various genes impelling early urethral development as well as genital tubercle may increase the risk of hypospadias [11]. Three genes of the AKR1C subfamily (*AKR1C2, AKR1C3*, and *AKR1C4*) as well as the *KLF6* gene were selected for mutation screening owing to their functioning in testosterone metabolism and expression in genital skin in hypospadias cases. These AKRs can convert potent sex hormones (androgens, estrogen, and progesterone) into their inactive metabolites by acting as 3-keto-, 17-keto-, and 20-ketosteroid reductases [10]. The male urethral development may be influenced by genistein through the means of alterations in pathways and disrupting genes in the mitogen-activated protein kinase (MAPK) and transforming growth factor-β (TGF-β) signaling pathways [12]. Gene expression in TGF-β and Wnt-Frizzled pathways has been found to be involved in the development of genital tubercle and urethral tube [13]. TGF-β is a potent regulator in the control of epithelial and endothelial cell proliferation, and this signaling pathway plays a critical role in the regulation of cell growth and differentiation, moreover, mutations which may affect the development and metastasis of cancer [14]. TGF-β functions in human cancers by means of a heteromeric receptor comprising TGF-β receptor type I (TGFBR1) and type II (TGFBR2), and genetic variations in TGFBR1 and TGFBR2 play an important role in pathogenesis of several diseases like gastric cancer and liver cancer [15]. Various researchers have demonstrated that mutations in the *TGFBR1* or *TGFBR2* genes lead to diseases such as colorectal cancer [16]. Additionally, heterozygous mutations in *TGFBR2* gene are commonly considered to be relative to the risk of Marfan syndrome, an autosomal dominant abnormality in connective tissues [17]. However, the roles of TGFBR1 or TGFBR2 gene polymorphisms in hypospadias have not yet been recorded. With regard to the diversity of gene polymorphism in different environments, the present study is designed to investigate the association of TGFBR1 and TGFBR2 gene polymorphisms with the risk of hypospadias in Chinese children.

## Materials and methods

### Ethics statement

This case–control study was carried out with the permission of the Ethics Committee of the Affiliated Municipal Hospital of Xuzhou Medical University and informed consent was received from the patients and their guardians.

### Study subjects

A total of 162 child patients with hypospadias who underwent urethroplasty in the Affiliated Municipal Hospital of Xuzhou Medical University from January 2014 to March 2015 were included in the case group with a calculated mean age of 4.54 ± 1.38 years. There was no blood relation amongst any of Han participants. Patients in the case group were divided into four subgroups according to the shape of fistula. There were 27 cases from coronary sulcus, 67 cases from penile coronary sulcus, 59 cases from penoscrotal junction coronary sulcus, and 9 cases from perineal coronary sulcus. The inclusion criteria for the study were as follows: (i) all patients were diagnosed as cases of isolated hypospadias at the Department of Urology, in which the urethra opens on to the ventral part of the penis, scrotum, or perineum; (ii) the opening position was manifested with ectopic urethral meatus, penile curvature, and accumulation of dorsal penile foreskin in these patients; (iii) patients did not have other genital deformities like hernia, hydrocele, or cryptorchidism. Meanwhile, 165 children who underwent circumcision in Department of Urology of the Affiliated Municipal Hospital of Xuzhou Medical University were selected as control group, with a calculated mean age of 4.35 ± 1.22 years. Children in the control group presented normal urethral opening, and were confirmed without other external genital deformities, such as hernia, hydrocele, or cryptorchidism. Baseline characteristics were recorded for further analysis including preterm birth (<37 weeks: preterm infants; 37–42 weeks: normal infants), infant birth weight (<2.5 kg was regarded as low birth weight infants; 2.5–4.0 kg were regarded as normal infants), abnormal pregnancy, medication during pregnancy, mother’s age at the time of pregnancy, and the number of prior pregnancies.

### SNP screening

The present study is based on the genomic data of Han population obtained from HapMap, and the SNPs of *TGFBR1* and *TGFBR2* genes were selected by literature review for Tag-SNPs, and Function Analysis and Selection Tool for SNPs (FASTSNP) analysis for TGFBR1 and TGFBR2 polymorphisms. Finally, TGFBR1 rs4743325 and TGFBR2 rs6785358 were considered as polymorphic loci in this analysis.

### Extraction of peripheral blood and genomic DNA

On day 2 post-admission, 5 ml of venous blood was collected from participants on an empty stomach and then placed in sodium citrate anticoagulant tube; and centrifuged at 3000 rpm for 10 min. The DNA from peripheral blood was extracted using a DNA Extraction Kit (item number: 52304, Qiagen, Hilden, Germany); the purity of DNA was measured using a DNA concentration detector (model: NanoDrop 2000, Thermo, Massachusetts, U.S.A.); DNA concentration was estimated by measuring the absorbance at 260 nm, adjusting the A260 measurement for turbidity (measured by absorbance at 320 nm), multiplying by the dilution factor, and using the relationship that A260 of 1.0 =50 µg/ml pure dsDNA. The average DNA concentration was 100 ± 20 ng/l, and the A260/A280 nm ratio was between 1.6 and 1.8. The extracted DNA was stored at –80°C.

### PCR-restriction fragment length polymorphism

PCR-restriction fragment length polymorphism (PCR-RFLP) was performed in order to detect TGFBR1 rs4743325 and TGFBR2 rs6785358 polymorphisms. Primers used in PCR-RFLP were designed using the Primer Premier 5.0 software and synthesized by the Shanghai Sangon Biological Engineering Technology & Services Co., Ltd. (Shanghai, China). The primer sequences and lengths are listed in Table 1. Each PCR reaction consisted of 1.5 μl of 10× PCR buffer, 0.3 μl dNTPs (deoxyribonucleoside triphosphates; 10 mmol/l), 0.25 μl forward primer (10 pmol/l), 0.25 μl reverse primer (10 pmol/μl), 0.25 μl Taq polymerase (5 U/μl; obtained from TaKaRa Biotechnology Co., Ltd., Dalian, China), and 1 μl DNA template (50 ng). In addition, sterile double-distilled water was added to maintain a constant volume of 15 μl. Reaction conditions were as follows: predenaturation at 94°C for 5 min, followed by 35 cycles of denaturation at 94°C for 30 s, annealing at 60°C for 30 s, and extension at 72°C for 30 s, and finally another round of extension at 72°C for 10 min. Negative control, in which the DNA template was substituted with sterile double-distilled water, added to each PCR reaction was run alongside to maintain the purity of the PCR system. A mixture of 3 µl PCR products and corresponding volume of 6× loading buffer was resolved by electrophoresis on a 3.5% agarose gel for 40 min at a voltage of 120 V. The solution was then stained with Ethidium Bromide (EtBr) and observed using a gel imaging system. Next, the PCR products were digested using a restriction enzyme. The reaction system (15 μl) included 6 μl PCR products, 1.5 μl of 10× enzyme digestion buffer and supplementary sterile double-distilled water to maintain a constant volume at 15 μl. The enzyme reaction was terminated after 16-h digestion in a 37°C water bath. A positive control, which selected a specific sequence containing these two cleavage sites, was set in every enzyme digestion to assure the accuracy of the system. Restriction enzymes HincII and BsuRI (TaKaRa Biotechnology Co., Ltd., Dalian, China) were used to identify the specific loci of digested PCR products (the working temperature of enzyme was 37°C, the concentration was 10 U/μl, and 0.2 μl of each enzyme was used in the experiment), and the genotype of digested PCR products was analyzed using a gel imaging system (Figure 1).

**Figure 1:** It is Gel imaging of the genotyping of rs4743325 and rs6785358 Gel imaging of the genotyping of rs4743325 (**A**) and rs6785358 (**B**). Abbreviation: M, marker.

**Table 1:** Primer sequences for PCR-RFLP

SNP	Primer sequence	Primer length
TGFBR1 rs4743325	F: 5′-GCCATTTTCTCCTCCACA-3′	256 bp
	R: 5′-CCAAAGGGCTCATCAAAG-3′	
TGFBR2 rs6785358	F: 5′-GAACTGCAAACAAGAGAATGGAT-3′	176 bp
	R: 5′-TTAGAATTCTACCCTAATGATTGTAAGG-3′	

Abbreviations: F, forward; R, reverse.

### Statistical analysis

Statistical analyses were performed using the SPSS software (version 19.0; SPSS Inc., Chicago, IL, U.S.A.). Chi-square goodness-of-fit test was applied in order to evaluate whether the genotype distributions in the two included groups meet Hardy–Weinberg equilibrium (HWE). The *t* test was employed for comparisons of clinical data between two groups. The genotype and allele frequencies between the case and control groups were compared. Genotype distribution and allele frequencies in the two included groups met the HWE. Logistic regression analysis was performed for risk-factor analysis, the results of which were presented as odds ratios (ORs), 95% confidence intervals (95% CIs). *P*<0.05 was considered to be statistically significant.

## Results

### Comparisons of clinical data between the case and control groups

Compared with the control group, there were high percentages of abnormal pregnancy and preterm birth in the case group. No significant differences in terms of low birth weight infant, medication during pregnancy, age at the time of pregnancy, and the number of prior pregnancies were observed between the case and control groups (all *P*>0.05) (Table 2).

**Table 2:** Comparisons of baseline characteristics between the case group and the control group

Characteristic	Case group (*n*=162)	Control group (*n*=165)	χ^2^/t	*P*
Age (years)	4.53 ± 1.43	4.35 ± 1.22	1.262	0.208
Preterm birth	22	6	10.320	0.001
Abnormal pregnancy	29	5	19.400	< 0.001
Low birth weight infant	15	8	2.432	0.119
Medication during pregnancy	9	2	4.744	0.029
Age at the time of pregnancy	28.18 ± 3.58	28.25 ± 4.06	0.165	0.869
Number of prior pregnancies	1.20 ± 0.44	1.15 ± 0.35	1.348	0.179

### Associations of TGFBR1 rs4743325 and TGFBR2 rs6785358 polymorphisms with hypospadias in a Chinese population

Genotype distribution and allele frequencies in the two included groups met the HWE. Genotype distributions as well as allele frequencies of TGFBR1 rs4743325 and TGFBR2 rs6785358 polymorphisms are shown in Table 3. The results revealed no significant difference in genotype distribution and allele frequencies of TGFBR1 rs4743325 polymorphism between the case and control groups (all *P*>0.05). However, genotype distributions and allele frequencies of TGFBR2 rs6785358 polymorphism in the case group were significantly different from those in the control group (all *P*<0.05). Subjects with the GA genotypes, AA genotypes, and GA + AA exhibited a significantly lower risk of congenital hypospadias compared with the GG genotype (GA compared with GG, OR =0.289, 95% CI =0.118–0.705, *P*=0.004; AA compared with GG, OR =0.120, 95% CI =0.050–0.287, *P*<0.001; GA + AA compared with AA, OR =0.173, 95% CI =0.074–0.405, *P*<0.001). Patients carrying the G allele exhibited an increased risk of hypospadias compared with the patients carrying the A allele in TGFBR2 rs6785358 (OR =2.931, 95% CI =2.063–4.165, *P*<0.001).

**Table 3:** Genotype distributions and allele frequencies of TGFBR1 rs4743325 and TGFBR2 rs6785358 polymorphisms in the case and control groups

Gene	Case (*n*=162)	Control (*n*=165)	OR (95% CI)	*P*
rs4743325				
TT	51 (31.48%)	48 (28.92%)	Ref.	
TG	79 (48.77%)	81 (48.8%)	0.917 (0.556–1.516)	0.738
GG	32 (19.75%)	36 (21.69%)	0.837 (0.451–1.553)	0.566
TG + GG	111 (68.52%)	117 (70.48%)	0.893 (0.557–1.432)	0.638
T	181 (55.86%)	177 (53.64%)	Ref.	
G	143 (44.14%)	153 (46.36%)	1.094 (0.804–1.489)	0.567
rs6785358				
GG	33 (20.37%)	7 (4.22%)	Ref.	
GA	68 (41.98%)	50 (30.12%)	0.289 (0.118–0.705)	0.004
AA	61 (37.65%)	108 (65.06%)	0.120 (0.050–0.287)	<0.001
GA + AA	129 (79.63%)	158 (95.18%)	0.173 (0.074–0.405)	<0.001
A	190 (58.64%)	266 (80.61%)	Ref.	
G	134 (41.36%)	64 (19.39%)	2.931 (2.063–4.165)	<0.001

Abbreviation: Ref., reference.

### Association of TGFBR1 rs4743325 and TGFBR2 rs6785358 polymorphisms with clinicopathological features of hypospadias

The clinicopathological features (age, abnormal pregnancy, preterm birth, low birth weight, medication during pregnancy, mother’s age at the time of pregnancy, and the number of prior pregnancies) of patients and genotype of TGFBR1 and TGFBR2 polymorphisms were studied and compared in the present study (Table 4). The TGFBR1 rs4743325 genotype demonstrated no significant association with age, preterm birth, abnormal pregnancy, low birth weight, medication during pregnancy, mother’s age at the time of pregnancy, and the number of prior pregnancies (all *P*>0.05). The TGFBR2 rs6785358 genotype was associated with abnormal pregnancy and preterm birth (*P*<0.05). The TGFBR2 rs6785358 genotype demonstrated no significant association with age, low birth weight, medication during pregnancy, mother’s age at the time of pregnancy, and the number of prior pregnancies (all *P*>0.05).

**Table 4:** Associations of TGFBR1 and TGFBR2 polymorphisms with clinicopathological features of patients with hypospadias

Feature	rs4743325			*P*-value	rs6785358			*P*-value
	TT	TG	GG		GG	GA	AA	
Age				0.984				0.397
>4 years old	25	40	16		14	38	29	
≤4 years old	26	39	16		19	30	32	
Preterm birth								0.008
Yes	6	9	7	0.311	5	3	14	
No	45	70	25		28	65	47	
Abnormal pregnancy			0.259				0.026	
Yes	6	18	5		1	17	11	
No	45	61	27		32	51	50	
Low birth weight infant				0.983				0.979
Yes	5	7	3		3	6	6	
No	46	72	29		30	62	55	
Medication during pregnancy				0.159				0.204
Yes	5	4	0		2	6	1	
No	46	75	32		31	62	60	
Age at the time of pregnancy				0.477				0.696
>28 years old	26	35	12		17	30	26	
≤28 years old	25	44	20		16	38	35	
The number of prior pregnancies				0.291				0.281
≤1	45	64	24		30	53	50	
>1	6	15	8		3	15	11	

### Associations of TGFBR1 rs4743325 and TGFBR2 rs6785358 polymorphisms with the pathological type of hypospadias

No significant differences were observed in the frequencies of three genotypes (TT/TG/GG) of the TGFBR1 rs4743325 polymorphism amongst patients suffering from four different pathological types of hypospadias (all *P*>0.05). However, significant differences were observed in the frequencies of TGFBR2 rs6785358 GG genotype amongst patients suffering from different types of hypospadias (*P*<0.05), implying that the GG genotype in TGFBR2 rs6785358 might be linked to the risk of hypospadias (Table 5).

**Table 5:** Associations of TGFBR1 rs4743325 and TGFBR2 rs6785358 polymorphisms with the pathological type of hypospadias

SNP	Coronary sulcus type *n*=27 (%)	Penile type *n*=67 (%)	Penoscrotal junction type *n*=59 (%)	Perineal type *n*=6 (%)	*P*
rs4743325					
TT	9 (33.33)	21 (31.34)	18 (30.51)	3 (33.33)	0.994
TG	14 (51.85)	32 (47.76)	29 (49.15)	4 (44.44)	0.978
GG	4 (14.81)	14 (20.90)	12 (20.34)	2 (22.22)	0.915
rs6785358					
GG	14 (51.85)	8 (11.94)	9 (15.25)	2 (22.22)	0.0001
GA	8 (29.63)	35 (52.24)	21 (35.59)	4 (44.44)	0.133
AA	5 (18.52)	24 (35.82)	29 (49.15)	3 (33.33)	0.053

### Multivariate logistic regression analysis of related risk factors for hypospadias

The risk of hypospadias was regarded as the dependent variable, while TGFBR2 rs6785358 polymorphism, preterm birth, abnormal pregnancy, low birth weight, medication during pregnancy, and the number of prior pregnancies served as independent variables in the logistic regression analysis. The findings revealed that preterm birth, abnormal pregnancy, and TGFBR2 rs6785358 polymorphism were the independent risk factors for hypospadias (*P*<0.05). Moreover, the TGFBR2 rs6785358 polymorphism might increase the risk of hypospadias 5.44-times (*P*<0.05) (Table 6).

**Table 6:** Logistic regression analysis of related risk factors for patients with hypospadias

Risk factor	OR	95% CI	*P*
Preterm birth	4.515	1.723–11.826	0.002
Abnormal pregnancy	5.238	1.883–14.567	0.002
TGFBR2 rs6785358 polymorphism	5.369	2.203–13.081	<0.001
Birth weight	2.195	0.857–5.623	0.102
Medication during pregnancy	4.954	0.989–24.816	0.052
Number of prior pregnancies	1.414	0.740–2.704	0.294

## Discussion

Hypospadias remains to be a common congenital abnormality in male external genitalia, with a mysterious etiology and challenging treatment regimens [18]. In this population-based study, we investigated the correlation of TGFBR1 and TGFBR2 gene polymorphisms with the risk of hypospadias in Chinese children, and reached a conclusion that TGFBR2 rs6785358 polymorphism may contribute to an increased risk of hypospadias.

Initially, the results revealed differences in the genotype and allele frequencies of TGFBR2 rs6785358 between the case and control groups, indicating that TGFBR2 rs6785358 may increase the risk of hypospadias. Changes in activity or levels of TGF-β are associated with a variety of diseases [19]. TGF-β is a multifunctional cytokine that mediates a diverse set of cellular activities such as cell proliferation, differentiation, as well as extracellular matrix deposition, and TGF-β coreceptors function by mediating the activity of TGF-β signaling in a cell-specific manner [20]. Mutations in the *TGFBR2* gene seem to be responsible for inactivation of the TGF-β pathway in colon cancer cells, which is a gene that encodes the TGF-β receptor, leading to abnormal cellular activities in colon cancer [21]. A recent study demonstrated that an injection of TGF-β1 into the urethral wall resulted in a urethral fibrosis-like condition in rats [22]. TGF-β1 is vital for prostatic smooth muscle regulation, as it induces the transdifferentiation of prostatic fibroblasts into myofibroblasts that secrete extracellular matrix components such as collagen and fibronectin [23]. Another study revealed that the expression of TGFBR2 affects the activation of TGF-β signaling in addition to involvement in the specific response of cells to TGF-β [24]. Evidence has revealed that mutations in genes affecting the reproductive tract development in males were found to carry some SNPs related to congenital abnormalities in the male genitalia [10,25]. Therefore, SNP rs6785358 in the *TGFBR2* gene which encodes different functions of the pathway may result in hypospadias by affecting the activity of TGF-β. Huang et al. [26] also reported that TGFBR2 rs6785358 are significantly linked to congenital heart defects in the Chinese male population.

Further analysis of the association amongst three genotypes (GA, AA, and GG) of TGFBR2 rs6785358 and the pathological type of hypospadias revealed statistical differences in the frequencies of GA or AA genotype, but not in the GG genotype, between the case and control groups. TGFBR2 rs6785358 polymorphism was reported to be correlated to the visceral leishmaniasis phenotype [27], which meant that TGFBR2 rs6785358 polymorphism was associated with the development of disease. The results of the present study also revealed that patients carrying a G allele of TGFBR2 rs6785358 might exhibit an increased risk of hypospadias. This result is similar to the finding of a recent study that demonstrated the G allele of TGFBR2 rs6785358 polymorphism may lead to a higher risk of congenital ventricular septal defect [28]. It is worth mentioning that the GG genotype produces a higher frequency of the least severe coronary sulcus disease.

Nonetheless, the present study revealed that the TGFBR1 rs4743325 SNP showed no association with hypospadias, implying that there was no correlation between SNP rs4743325 in TGFBR1 and hypospadias. However, we could not reach a conclusion that TGFBR1 is not related to hypospadias. Evidence demonstrated the presence of high frequency of TGFBR1 allele-specific expression phenotype in non-small-cell lung cancer tumors [29]. Germline allele-specific expression of TGFBR1 is more likely to result in an increased risk of colorectal cancer [30]. Besides, a previous meta-analysis revealed that the TGFBR1*6A/9A polymorphism is susceptive to cancer, increasing the risk of breast and ovarian cancers [31]. Logistic regression analysis indicated that preterm births, abnormal pregnancy, and TGFBR2 rs6785358 polymorphism were independent risk factors for hypospadias. In addition, the genotype of TGFBR2 rs6785358 was significantly related to abnormal pregnancy and preterm birth. A multifactorial etiology has been reported in hypospadias, which is an interaction of both genetic and environmental factors [25]. The results showed that various factors are related with hypospadias, which was consistent with the report of Manson et al. [32] stating that paternal subfertility, familial clustering, intrauterine growth reduction, genes involved in androgen activity, and gene pathways were risk factors for hypospadias. Here, the TGFBR2 rs6785358 polymorphism has a risk factor of hypospadias, which would provide an evidence for the potential diagnostic value.

In summary, the present study showed that SNP rs6785358 of TGFBR2 might increase the risk of hypospadias, but SNP rs4743325 of TGFBR1 exhibited no significant association with hypospadias in this Han-Chinese cohort study. These results imply that TGFBR2 rs6785358 polymorphisms may be used as a biological predictor during the early diagnosis of hypospadias. However, there are some limitations of our study. First, the sample size of the study was relatively small. Second, our study only focussed on a Chinese population. Therefore, further investigations including a larger sample size of different ethnic groups are required to confirm our findings. Additionally, molecular mechanisms of this genetic predisposition should be investigated in the future.

## Abbreviations

BMI: body mass index
HWE: Hardy–Weinberg equilibrium
OR: odds ratio
PCR-RFLP: PCR-restriction fragment length polymorphism
SNP: single nucleotide polymorphism
TGFBR1: transforming growth factor-β receptor type I
TGFBR2: transforming growth factor-β receptor type II
TGF-β: transforming growth factor-β
95% CI: 95% confidence interval
